This article has been retracted.

# Butein inhibits metastatic behavior in mouse melanoma cells through VEGF expression and translation-dependent signaling pathway regulation

**DOI:** 10.1186/s12906-015-0970-3

**Published:** 2015-12-22

**Authors:** Yu-Wei Lai, Shih-Wei Wang, Chien-Hsin Chang, Shih-Chia Liu, Yu-Jen Chen, Chih-Wen Chi, Li-Pin Chiu, Shiou-Sheng Chen, Allen W. Chiu, Ching-Hu Chung

**Affiliations:** Department of Urology, National Yang-Ming University School of Medicine, Taipei, Taiwan; Division of Urology, Taipei City Hospital Renai Branch, Taipei, Taiwan; Department of Medicine, Mackay Medical College, No. 46, Sec. 3, Jhong-Jheng Rd., Sanzhi Dist., Taipei, Taiwan; Institute of Pharmacology, College of Medicine, National Taiwan University, Taipei, Taiwan; Department of Orthopaedics, Mackay Memorial Hospital, Taipei, Taiwan; Department of Medical Research, Mackay Memorial Hospital, Taipei, Taiwan; Department of Radiation Oncology, Mackay Memorial Hospital, Taipei, Taiwan

**Keywords:** Melanoma, Butein, Mammalian target of rapamycin, Metastasis, Vascular endothelial growth factor, mTOR, VEGF

## Abstract

**Background:**

Melanoma is an aggressive skin cancer and a predominant cause of skin cancer-related deaths. A previous study has demonstrated the ability of butein to inhibit tumor proliferation and invasion. However, the anti-metastatic mechanisms and in vivo effects of butein have not been fully elucidated.

**Methods:**

MTT cell viability assays were used to evaluate the antitumor effects of butein in vitro. Cytotoxic effects of butein were measured by lactate dehydrogenase assay. Anti-migratory effects of butein were evaluated by two-dimensional scratch and transwell migration assays. Signaling transduction and VEGF-releasing assays were measured by Western blotting and ELISA. We also conducted an experimental analysis of the metastatic potential of tumor cells injected into the tail vein of C57BL/6 mice.

**Results:**

We first demonstrated the effect of butein on cell viability at non-cytotoxic concentrations (1, 3, and 10 μM). In vitro, butein was found to inhibit the migration of B16F10 cells in a concentration-dependent manner using transwell and scratch assays. Butein had a dose-dependent effect on focal adhesion kinase, Akt, and ERK phosphorylation in B16F10 cells. Butein efficiently inhibited the mTOR/p70S6K translational inhibition machinery and decreased the production of VEGF in B16F10 cells. Furthermore, the in vivo antitumor effects of butein were demonstrated using a pulmonary metastasis model.

**Conclusion:**

The results of the present study indicate the potential utility of butein in the treatment of melanoma.

## Background

The incidence of melanoma of the skin has rapidly increased in recent years and is currently the most common fatal form of skin cancer [1]. New Zealand has the highest incidence of invasive melanoma worldwide with an age-standardized rate of 40.2/100,000 [2]. Asian populations, including China, India, Japan, and Singapore, are reported to have relatively lower incidence rates (approximately 1/100,000). Despite being a relatively rare cancer, melanoma is associated with substantial morbidity and mortality. This notorious aggressiveness of melanoma is associated with its metastatic propensity, which can occur even from shallow primary tumors [3]. According to the clinical evidence, the survival rate in patients with multiple site of metastasis disease is less than 5 % [4]. Despite significant progress in understanding the biology of melanoma, new targets and immune-modulatory therapies (such as vermurafenib and ipilimumab) have demonstrated efficacy in improving the overall survival in melanoma patients [5, 6]. However, the benefit of these therapies is variable, and tumor metastasis still occurs in majority of the melanoma patients.

Surgery is the most important treatment for malignant melanoma. However, late stage and metastatic melanoma is known to confer a very poor prognosis, with no standard of care currently established. Drug therapies for melanoma, including chemotherapy and targeted therapy, are currently under development. The pathogenesis of melanoma is complex and involves a number of signaling pathways related to tumor cell growth and metastasis [7]. Up-regulation of the mitogen activated protein kinase (MAPK) signaling pathway is common in many human cancers, including melanoma [8]. The phosphatidylinositol 3-kinase (PI3K)/Akt signaling pathway represents another key mediator of these processes. PI3K can activate Akt and subsequently phosphorylate several target proteins, including mammalian target of rapamycin (mTOR). Following mTOR activation, cell growth promotion and cell cycle progression may occur because of mTOR downstream p70S6 kinase (p70S6K) and eukaryotic initiation factor (eIF) 4E-binding protein 1 (4E-BP1) phosphorylation [9, 10]. The MAPK and PI3K/Akt/mTOR signaling pathways are frequently activated and dysregulated in melanoma, and both represent promising targets for melanoma treatment. Agents that target the MAPK signaling pathway (AS/RAF/MEK/ERK), such as vemurafenib (a BRAF inhibitor) and trametinib (a MEK1/2 inhibitor), have increased survival in patients with metastatic melanoma [11]. Inhibition of the Akt/mTOR signaling pathway has also been shown to abolish invasion and metastasis of highly-metastatic melanoma cells [12]. MAPK and Akt/mTOR signaling pathway inhibitors may represent promising targets for the inhibition of melanoma cell invasion and metastasis.

Butein (3,4,2′,4′ -tetrahydroxychalcone) is a flavonoid and chalcone derivative [13]. Flavonoids are phenolic agents used in traditional Chinese and Tibetan herbal medicines, which can be extracted from numerous plant tissues, including the stem bark of cashews (*Semecarpus anacardium*), the heartwood of *Dalbergia odorifera*, and *Caragana jubata* and *Rhus verniciflua* stokes. Butein has been found to have anti-oxidant, anti-inflammatory, and anti-restenosis activities, which may be beneficial in disease treatment [14–16]. Recent studies have reported that butein exhibits anti-angiogenesis, anti-proliferation, and apoptotic effects against numerous cancer cell lines [17–19]. In our previous study, we demonstrated that butein significantly inhibited invasion of SK-Hep-1 cells, a hepatoma cell line, via Akt/mTOR/p70S6K blockade [20]. However, the effects of butein on tumor metastasis are yet to be determined. Thus, we hypothesized that butein has a similar inhibitory effect on Akt/mTOR/p70S6K signaling pathway and the proliferation and metastasis of melanoma cells. In the present study, we aimed to elucidate the mechanisms underlying the anti-metastatic effect of butein. We found that butein diminished the PI3K/Akt/mTOR signaling pathway in the mouse melanoma cell line, B16F10. In addition, butein demonstrated potent anti-metastatic effects in a model of lung metastasis.

## Methods

### Materials

2',3,4,4'-Tetrahydroxychalcone (butein) was purchased from Extrasynthese Corporation (Genay, France). Dulbecco's Modified Eagle Medium (DMEM), fetal bovine serum (FBS), Antibiotic-Antimycotic and trypsin-EDTA were purchased from Gibco (Grand Island, NY). Toluidine blue O, RNase A and 3-[4,5-dimethylthiahiazo-2-y1]-2,4-diphenytetrazolium bromide (MTT) were purchased from Sigma Chemical Corporation (St Louis, MO, U.S.A.). Lactate dehydrogenase (LDH) assay reagents were purchased from Promega Corporation (Madison, WI). Antibodies for phospho-Akt (Ser473), phospho-mTOR (Ser2448) were purchased from Epitomics (Burlingame, CA). Antibodies for phospho-ERK1/2 (Thr202/Tyr204), phospho-p70S6K (Thr389) and α-tubulin were purchased from Cell Signaling Technologies (Boston, MA).

### Cell culture

Mouse melanoma cells (B16F10) were obtained from the American Type Culture Collection. B16F10 cells were cultured at 37 °C in HEPES-buffered Dulbecco’s modified Eagle’s medium (DMEM), containing 10 % fetal bovine serum (Gibco) supplemented with NaHCO3, glutamax I (Gibco), 100 IU/mL penicillin G (sodium salt), 100 μg/mL streptomycin and 0.25 μg/mL amphotericin B (antibiotic-antimitotic solution, Gibco).

### Cell viability assay

B16F10 cells were sub-cultured onto 24-well plates and starved with serum-free DMEM for 48 hours. Then, melanoma cells were grown in DMEM, included 10 % FBS in absence or presence of various concentrations of butein (1, 3, 10 μM) for 48 hours. Cells were incubated with MTT (0.5 mg/mL) for 4 hours. Formazan crystal (purple) was lysed by dimethyl sulfoxide (DMSO) and absorbance was measured at 550 nm with ELISA-reader (Thermo, U.S.A.).

### Lactate Dehydrogenase Assay

B16F10 cells were seeded onto 48-well plates in a density of 2 × 10^4^ cells/well and starvation for 48 hours with serum-free DMEM and incubated with or without vehicle and indicated concentrations of butein (1, 3 and 10 μM) in DMEM with 10 % FBS. The percentage of LDH release was calculated from the ratio of LDH activity in the medium to LDH activity in the cell lysate.

### Migration assay

Migration assay of B16F10 cells was measured by Coaster Transwells (polycarbonate filter, 8 μm pore size) which were coated with 0.2 % gelatin. B16F10 cells (5x10^4^cell/well) were treated with vehicle or various concentrations of butein (1, 3, 10 μM), and then cells were seeded into the upper chamber. The bottom chamber was added DMEM medium supplemented with 10 % FBS. After incubation at 37 °C for 16 hr, all non-migrant cells were removed from the upper face of the Transwell membrane with a cotton swab, and the B16F10 cells that had transmigrated through the micropore and that were still bound to the membrane were fixed with 4 % paraformadehyde in PBS solution and stained with 0.5 % toluidine blue in 4 % paraformadehyde. Migration was quantified by counting the number of stained cells on the membrane under a light microscope (Nikon, Japan) at a magnification of 200× in 3 random fields, and then photographed. All determinations were obtained by replication in at least three independent experiments.

### Two-dimensional Migration Scratch Assay

Sub-cultured B16F10 cells were seeded into 6-well plates. B16F10 cells were starved with serum-free DMEM for 48 hours. Part of the dish was denuded by scratching along a straight line with a 200 μl pipet tip and incubated with or without vehicle and indicated concentrations of butein (1, 3 and 10 μM) in DMEM with 10 % FBS. After 16 hours of incubation at 37 °C, images of the wounded area were captured immediately by microscope (Nikon, Japan).

### Western blotting

After cells pretreated with or without various concentrations of butein (1, 3, 10 μM) and vehicle in serum-free DMEM for 2 hours, cells were harvested and lysed in a lysis buffer containing 15 mM Tris–HCl, 50 mM NaCl, 5 mM EGTA (ethyleneglycoltetraacetic acid), 1 % Triton X-100, 1 % sodium deoxycholate, 0.1 % sodium dodecyl sulfate (SDS), 1 mM NaF, 1 mM phenylmethylsulfonyl fluoride (PMSF), 1 mM Na_3_VO_4_, 10 μg/mL aprotinin, and 10 μg/mL leupeptin, pH 7.4. The protein samples separated on 10 % SDS-PAGE were then transferred to PVDF membranes by electro-blotting. The membranes were blocked with 0.25 % (wt/vol) gelatin at room temperature 1 hour. Afterward, immune-detection for phosphorylated (activated) FAK, Akt, ERK, mTor, p70S6K, eIF4E and α-tubulin were accomplished with antibody in 0.25 % (wt/vol) gelatin. Blots were washed for at least 30 mins in wash buffer (Tris/phosphate/saline/Tween). After incubation with each antibody, the immunoreactive band was detected by an Enhanced Chemiluminiscence (ECL) Western blotting detection system.

### ELISA

B16F10 cells (10^5^cells/well in 96well) were treated with various concentrations of Butein or vehicle for 24 hr, and then the supernatant was collected to examine the amount of vascular endothelial growth factor (VEGF) protein. VEGF mouse ELISA Kit (Novex®, Invitrogen) was used according to the manufacturer’s instructions.

### Animals

8-10 weeks-old male C57BL/6 mice were used in all studies. All the experimental protocols regarding animal study have been approved by the Institutional Animal Care and Use Committee at College of Medicine, Tzu-Chi University.

### Experimental metastasis analysis

Metastasis analysis was performed as previously described [21]. Briefly, B16F10 cells (2 × 10^6^ cells) were slowly injected into the lateral tail vein of C57BL/6 mouse to initiate tumor metastasis. Butein (1、3、10 mg/kg) was intraperitoneally administered to mice every day from 3 days before tumor cell injection to 21 days after tumor cell injection (the day sacrified).

### Statistical analysis

All values are presented as mean ± SEM. Differences between groups were assessed by one-way ANOVA and Newman–Keuls multiple comparison test where appropriate. P values less than 0.05 (P < 0.05) were considered to be significantly different.

## Results

### Effects of butein on the inhibition of B16F10 melanoma proliferation

The structure of butein is shown in Fig. 1a. The effects of butein on melanoma cell proliferation were determined by MTT assay. As shown in Fig. 1b, butein inhibited B16F10 proliferation in a concentration-dependent manner (IC50 = 9.53 μM). To confirm that the anti-proliferative effect of butein was not because of cytotoxicity, an LDH assay was also performed. Our data indicates that butein does not have cytotoxic effects on B16F10 cells at a concentration of 10 μM (Fig. 1c).

**Fig. 1:** The structure of butein and its effect on melanoma cells viability and cytotoxicity. The structure of butein is shown in **a**. B16F10 cells were seeded onto plates for 24 hr and starved for another 24 hr with serum-free DMEM. **b** Quiescent cells were cultivated with DMEM containing 10 % FBS in the absence or presence of various concentrations of butein. After 48 h, cell viability was detected by the MTT assay. **c** Cytotoxicity was detected by manufacture’s protocol and finally recorded absorbance at 490 nm. Control was taken as basal condition of LDH release. The results are presented as percentages of inhibition (mean ± SEM, *n* = 4). All *P* values were obtained from comparisons between control and indicated concentration-treated cells. **, *P* < 0.01; ***, *P* < 0.001

### Butein inhibits serum-stimulated cell motility

Migration is a major step in melanoma metastasis. The pre-treatment addition of various concentrations of butein (1, 3, and 10 μM) to the upper wells of transwell chamber significantly inhibited B16F10s migration in response to 10 % FBS (Fig. 2a). Furthermore, we produced scrape wounds on B16F10 monolayers to observe the continuous movement of B16F10 cells in closing the gap that was denuded. After 16 h of continuous treatment, butein (1, 3, and 10 μM) inhibited the serum-stimulated cell motility of melanoma cells (Fig. 3a). Migration responses of melanoma cells in both modified Boyden chamber assays and scrape models were significantly reduced in a concentration-dependent manner.

**Fig. 2:** Effect of butein on serum-stimulated B16F10 cell migration. **a** B16F10 cells (2 × 10^4^) cultured in serum-free DMEM were pretreated with or without butein for 30 minutes, and placed in the upper chamber of a Transwell containing with 0.2 % gelatin-coated filter membrane. DMEM with 10 % FBS was added to the lower chamber. After removal of non-migrated cells and fixation, cells that migrated to the underside filter membrane were stained and quantified by phase-contrast light microscope under a high-power field (HPF; magnification, 100×). Three fields per filter were counted at 100× magnification. The quantitative of migratory cell was shown in **b**. Data are expressed as mean ± S.E.M. of five independent experiments. *p < 0.05; **p < 0.01 compare with the control (Veh) group

**Fig. 3:** Effect of butein on serum-stimulated B16F10 cell motility. **a** B16F10 cells (5 × 10^4^) were seeded onto 6-well plates for 24 hr and starved for another 24 hr with serum-free DMEM. Cells were subjected to injury by scratching with a plastic pipette tip (200 μl). The cells were then treated for 24 hours with or without serum or butein. The quantitative of migratory cell was shown in **b**. Data are presented as percentages of control (mean ± S.E.M., n = 3). **, *P* < 0.01 and ***,*P* < 0.001 versus control group

### Butein inhibits the ERK, focal adhesion kinase (FAK), and PI3K/Akt/mTOR/p70S6K signaling pathways in melanoma cells

The MAPK and PI3K/Akt/mTOR signaling pathways are well-known important signaling pathways for melanoma growth and metastasis. Follow-up experiments were designed to determine the effect of butein on signaling-related protein phosphorylation in B16F10 cells. Butein dramatically inhibited Akt and ERK1/2 phosphorylation in a concentration-dependent manner in B16F10 cells. mTOR, an important downstream effector of the PI3K/Akt signaling pathway, is known to regulate translational-related processes via stimulation of p70S6K and 4EBP1 phosphorylation. Thus, we evaluated the effects of butein in the modulation of these signaling pathways. As shown in Fig. 4a, serum (10 % FBS) induced a significant increase in mTOR, p70S6K, 4E-BP1, and eIF4E phosphorylation. In response to the serum, mTOR phosphorylation and major downstream targets, including p70S6K, 4EBP, and eIF4E, were significantly attenuated by butein treatment in a concentration-dependent manner. The FAK-mediated signaling cascade has also been shown to be involved in melanoma migration and mitogenic responses [22]. Accordingly, we further assessed the effect of butein on FAK phosphorylation. We observed that the levels of serum-induced FAK phosphorylation were also inhibited by butein. These results indicate that butein may inhibit B16F10 growth and migration through the inhibition of cellular signaling pathways.

**Fig. 4:** Effect of butein on PI3K/Akt/mTOR, ERK and FAK pathways. **a** B16F10 cells were incubated in the absence or presence of butein (1- to 10 μM) for 12 hrs. Then, the cells were harvested and lysed for the detection of the PI3K/Akt/mTOR, ERK and FAK pathways activation by Western blot. The quantitative densitometry of the relative level of protein phosphorylation (phosphortlation protein/total protein) was performed with Image-Pro Plus and was shown in **b**. Data are expressed as mean ± S.E.M. of five independent experiments. The protein phosphorylation in all treatment cells were significant lower than control (Veh) group (***p < 0.001 as compare with control (Veh) group)

### Butein inhibits VEGF release

The expression and production of VEGF is regulated by downstream transcript factors of the PI3K/Akt/mTOR signaling pathway. Therefore, we examined the effect of butein on VEGF release in B16F10 cells. After 24-h treatment with various concentrations of butein, supernatants were collected for analysis. VEGF release was found to be suppressed by butein in a concentration-dependent manner in B16F10 cells (Fig. 5).

**Fig. 5:** Effects of butein on VEGF production in melanoma cells, B16F10. VEGF protein expression was evaluated by ELISA in conditioned medium of B16F10 in the presence or absence of butein at the indicated concentrations. Data are represented as mean ± SEM (n = 6). *P < 0.05 and **P < 0.01 indicates significant differences from the vehicle control

### Butein inhibits in vivo pulmonary metastasis in B16F10 cells

As the migration activity of B16F10 cells is associated with tumor metastasis, we investigated the in vivo effect of butein in a murine pulmonary metastasis model. Single intravenous bolus injections of 2 × 10^6^ B16F10 cells were used to induce lung metastases. Butein (1, 3, or 10 mg/kg) was intraperitoneally administered to mice from 3 days before tumor cell injection. Twenty-one days later, the mice were euthanized, and their lungs were removed. Mice treated with butein were found to have a significant dose-dependent reduction in lung metastases (Fig. 6a). The quantitative of lung metastasis colony was shown in Fig. 6b. Butein significantly attenuated pulmonary metastasis of B16F10 cells in vivo.

**Fig. 6:** Effects of butein on experimental lung metastasis. **a** B16F10 cells (2x10^6^) were injected into the lateral tail vein of C57BL/6 mouse. Twenty days later, the lungs were removed, and surface-visible tumors were counted in the absence and presence of butein treatment. The melanoma metastasis area of lung surface was black and background is dark red. White area was quantified using ImageJ software. The quantitative of lung metastasis colony was shown in **b**. Corresponding bar graph expressed as percentage of vehicle (n = 8)

## Discussion

Metastasis is a deadly stage in cancer progression and the also is an important prerequisite for cancer metastasis [23, 24]. There remains a lack of promising therapeutic agents for the prevention of melanoma invasion and metastasis. The results of the present study demonstrated that a naturally occurring chalcone derivative, butein, significantly inhibited melanoma proliferation and migration in a concentration-dependent manner (1, 3, and 10 μM) without significant cytotoxicity (Fig. 1b, c). We previously reported that butein has anti-metastatic activity by reducing MMP-9/uPA proteolytic and Akt/mTOR/p70S6K translational activity [20]. In the present study, butein treatment for 16 h was found to inhibit cell migration at concentrations ranging from 1 to 10 μM. Under similar conditions, butein was found to induce substantial amounts of cell death at a concentration of 10 μM only. These data indicate that the migration inhibitory effect of butein is not because of cytotoxicity. To the best of our knowledge the present study is the first to provide evidence of the inhibitory effects of butein on melanoma metastasis, without showing a significant effect on cell proliferation. We demonstrated that butein exhibited anti-metastatic activity at low concentrations (1 μM) without inducing significant cell death in B16F10 cells. Notably, we also found that butein significantly attenuated pulmonary metastasis of B16F10 cells in vivo (Fig. 6). We also summarize the contents and major findings in Fig. 7.

**Fig. 7:** Schematic presentation of butein-mediated signaling transduction modulation

Dysregulation of the PI3K/Akt/mTOR signaling pathway has been observed in various human cancers. As the PI3K/Akt/mTOR signaling pathway regulates various important cellular processes, it has become an most important therapeutic targets for anti-cancer drug development [9, 10, 25]. The mTOR signaling pathway is a major chemotherapy target for the treatment of cancers, including melanoma [11]. We found that mTOR phosphorylation, its upstream kinases, PI3K, Akt, and the downstream effector, p70S6K, in B16F10 cells (Fig. 4) were all effectively inhibited by butein. The mTOR signaling pathway is also regulated by PI3K/Akt-independent signaling pathways, such as ERK, p38 MAPK, and AMPK [26]. FAK has been shown to be important for melanoma cell proliferation, adhesion, and invasion in vitro and in vivo [27]. FAK inactivation reportedly results in decreased ERK phosphorylation and VEGF expression [22]. These studies have demonstrated that FAK plays a critical role in melanoma metastasis and may represent an anti-metastatic target for melanoma treatment. As butein also significantly inhibited the FAK and ERK signaling pathways, the anti-cancer effect of butein may also be dependent on the inhibition of the FAK and ERK signaling pathways.

Activation of mTOR via the PI3K/Akt signaling pathway is associated with increased translation of hypoxia-inducible factor (HIF)-1α, which drives the expression of angiogenic growth factors [28]. As butein was found to inhibit mTOR activation, we hypothesize that butein may suppress VEGF gene expression in B16F10 cells. Previous studies have reported that aggressive melanoma cell lines express higher levels of VEGF and that melanoma patients with higher VEGF concentrations have a higher rate of relapse [29, 30]. Inhibition of tumor growth has been achieved in different melanoma xenograft models through the use of a number of anti-VEGF strategies [31]. In the present study, VEGF production was decreased in B16F10 cells after 24-h treatment with butein in a concentration-dependent manner (Fig. 5). VEGF production has also been reported to be associated with activation of downstream signaling pathways and phenotypic changes, such as increased cell migration and invasion [32]. Furthermore, VEGF expression has been reported to have a correlation with apoptosis, and VEGF reduces cell death through an autocrine mechanism [33, 34]. The inhibitory effect of butein on VEGF expression may induce apoptosis of B16F10 cells in addition to reducing tumor metastasis.

Surgery remains the major treatment for malignant melanoma. However, the prognosis of melanoma remains poor because of the invasiveness and metastasis of the tumors [35]. Therefore, more efficacious treatments for melanoma metastasis are required. Butein reduced the number of lung metastasis foci in a dose-dependent manner in an in vivo pulmonary metastasis model, indicating the anti-metastatic and antitumor activities of butein towards melanoma (Fig. 6).

There are still some limitations in this study. According to the Flaherty *et al*. study, approximately 50 % of melanomas harbor activating BRAF mutations [36]. Human melanomas display abnormal activation of the MAPK cascade due to these mutations and may exhibit sensitivity to MEK inhibition. Although the mouse melanoma cell, B16F10, were without mutations in the BRAF and NRAS genes, the MAPK cascade and PI3K/Akt signaling pathway are still the major mediators for melanoma metastasis. So far, the best characterized of metastasis models is the B16 melanoma model. B16F10 cells had an effective metastasis rate of 5 × 10^-5^ per cell per generation [37]. Beside human melanoma cell transplanted null mice, this metastasis model in conjunction with in vitro modeling and manipulation of tumor cells have enable investigators to development of agents that can be used to prevent or treat overt metastatic disease.

## Conclusion

We demonstrated that butein inhibits tumor growth in vitro by inhibiting the ERK and PI3K/Akt/mTOR signaling pathways. VEGF production was found to be decreased following butein treatment. More importantly, butein exhibited anti-tumor activity by in vivo pulmonary metastasis model. Collectively, the results of the present study indicate that butein has potential anti-cancer properties for the treatment of melanoma. However, clinical trials are required to fully validate the potential of butein in clinical applications.

## Abbreviations

PI3K: phosphatidylinositol 3-kinase
mTOR: mammalian target of rapamycin
p70S6K: p70S6 kinase
VEGF: vascular endothelial growth factor
